# Comparative proteomic analysis reveals the regulatory network of the *veA* gene during asexual and sexual spore development of *Aspergillus cristatus*

This article has been retracted.

**DOI:** 10.1042/BSR20180067

**Published:** 2018-07-31

**Authors:** Hui Liu, Shilei Sang, Hui Wang, Xiyi Ren, Yumei Tan, Wei Chen, Zuoyi Liu, Yongxiang Liu

**Affiliations:** 1 Guizhou Biotechnology Institute, Guizhou Academy of Agricultural Sciences, Guiyang, Guizhou 550006, China; 2 Guizhou Key Laboratory of Agricultural Biotechnology, Guiyang, Guizhou 550006, China; 3 Institute of Groundwater and Earth Sciences, Jinan University, Guangzhou 510632, China; 4 School of Life Science, Shanxi Normal University, Linfen 041000, Shanxi, China

**Keywords:** ascospore, Aspergillus cristatus, conidia, proteomics, veA gene

## Abstract

*Aspergillus cristatus* is the predominant fungal population during fermentation of Chinese Fuzhuan brick tea, and belongs to the homothallic fungal group that undergoes a sexual stage without asexual conidiation under hypotonic conditions, while hypertonic medium induces initiation of the asexual stage and completely blocks sexual development. However, the *veA* deletion mutant only produces conidia in hypotonic medium after a 24-h culture, but both asexual and sexual spores are observed after 72 h. The *veA* gene is one of the key genes that positively regulates sexual and negatively regulates asexual development in *A. cristatus*. To elucidate the molecular mechanism of how VeA regulates asexual and sexual spore development in *A. cristatus*, 2D electrophoresis (2-DE) combined with MALDI-tandem ToF MS analysis were applied to identify 173 differentially expressed proteins (DEPs) by comparing the agamotype (24 h) and teleomorph (72 h) with wild-type (WT) *A. cristatus* strains. Further analysis revealed that the changed expression pattern of Pmk1-MAPK and Ser/Thr phosphatase signaling, heat shock protein (Hsp) 90 (HSP90), protein degradation associated, sulphur-containing amino acid biosynthesis associated, valine, leucine, isoleucine, and arginine biosynthesis involved, CYP450 and cytoskeletal formation associated proteins were involved in the production of conidia in agamotype of *A. cristatus*. Furthermore, the deletion of *veA* in *A. cristatus* resulted in disturbed process of transcription, translation, protein folding, amino acid metabolism, and secondary metabolism. The carbohydrate and energy metabolism were also greatly changed, which lied in the suppression of anabolism through pentose phosphate pathway (PPP) but promotion of catabolism through glycolysis and tricarboxylic acid (TCA) cycle. The energy compounds produced in the agamotype were mainly ATP and NADH, whereas they were NADPH and FAD in the teleomorph. These results will contribute to the existing knowledge on the complex role of VeA in the regulation of spore development in *Aspergillus* and provide a framework for functional investigations on the identified proteins.

## Introduction

Fuzhuan brick tea is a dark tea with a history of over 400 years and is prevalent in China and Northeastern Asia [1]. Microbial fermentation exerts a critical role in the organoleptic qualities and health properties of Fuzhuan brick tea. Various fungal taxa participate in this fermentation, including *Aspergillus, Eurotium*, and *Penicillium* species, and *Aspergillus cristatus* is dominant [2]. The yellow cleistothecium of *A. cristatus* constitutes the ‘Golden Flower’ [3].

Spore gender is determined according to growth conditions [4]. Osmotic pressure (hypotonic/hypertonic conditions) plays a critical role in *A. cristatus* sporogenesis. *A. cristatus* grown on hypo-osmolar medium only reproduces sexually, but only asexual conidia are produced in ≥3 M NaCl conditions, where sexual reproduction is totally inhibited [5]. However, in the present study, the *veA* deletion mutant reproduced asexually only after 24 h of culture in hypo-osmolar medium, whereas both asexual and sexual spores were produced after 72 h (Figure 1). Similarly, sexual reproduction in the *veA1* mutants of *A. nidulans, A. parasiticus, A. xavus, Fusarium verticillioides*, and *Neurospora crassa* are generally retarded and reduced, while asexual development is promoted and increased [6–8], indicating that VeA positively regulates sexual development but negatively modulates asexual development in these filamentous fungal species.

**Figure 1:** Optical micrographs of the wild-type (WT) and *ΔveA* deletion-type *A. cristatus* strains (**A**) Optical micrograph of WT *A. cristatus* strains under low osmotic pressure; (**B**,**C**) optical micrograph of the Δ*veA* deletion-type *A. cristatus* strains under low osmotic pressure at 24 and 72 h, respectively. (**a**) The structure of ascospores detected in (A); (**b**) the conidia detected in (B) with developing metulae; (**c**,**d**) were the single mature ascospores and conidia observed in (C), respectively.

A molecular functional analysis of VeA in the model fungus *A. nidulans* revealed that VeA is transported to the nucleus by the α-importin KapA, where it interacts with LaeA, FphA, LreA, LreB, and VelB to form a regulatory complex that regulates the expression of spore development-associated genes [9]. An *Aspergillus* transcriptome analysis revealed that VeA regulates the expression of hundreds of genes [10], including additional roles in hydrolytic activity and the oxidative stress response [11], toxin and sclerotial production [8], and production of gliotoxin, proteases [12], and secondary metabolites [13–15]. However, the underlying mechanisms are not fully understood despite the abundance of information on the *veA* functional regulatory system provided by deletion mutants, protein–protein interaction studies, and genomics analyses because the VeA protein does not share homology with other proteins with a known function [13]. Furthermore, knockdown of the *veA* gene in *A. fumigatus* reduces conidia sporulation rather than enhance asexual conidia production in other *Aspergillus* species, and overexpression of this gene further reduces conidial production [12], suggesting that different *Aspergillus* species respond to the *veA* deletion differently. Therefore, a comparative proteomics analysis was applied in the present study to interpret the *A. cristatus* molecular regulatory mechanisms rendered by VeA.

Comparative proteomics analysis is a powerful method that offers qualitative and quantitative expression profiling of all proteins and furthers the systematic understanding of molecular events after a functional analysis of the identified proteins [16]. 2D electrophoresis (2-DE) is one of the most frequently used and powerful techniques applied to separate proteins [17]. Various virulence factors, diagnostic markers, and environmental stress response-associated proteins have been identified in fungi using proteomics analysis [16,18]. To understand the regulatory mechanisms of the VeA protein during spore development in *A. cristatus*, we employed 2-DE to study system-wide protein expression regulated by VeA. We found that the majority of proteins affected were involved in genetic information processes, carbon metabolism, energy metabolism, and secondary and amino acid metabolism. Our results indicate that the VeA protein regulates complex metabolism in *A. cristatus*.

## Materials and methods

### Fungal strains, culture medium, and growth conditions

The wild-type (WT) *A. cristatus* strain used in the present study was GZAAS20.1005 (isolated from Fuzhuan brick tea by single spore isolation), provided by the Key Laboratory of Guizhou Agricultural Biotechnology (Guiyang, China). Genetically stable *ΔveA* knockout strains (deletion-type) were constructed by our lab previously [19].

A low osmotic pressure malt extract (MYA) medium was applied for strain culture and contained 20 g malt extract, 30 g sucrose, 5 g yeast extract powder, 15 g agar (not in the liquid medium), 1 M NaCl, and 1000 ml double distilled water.

The ascospore solution of the WT and deletion-type *A. cristatus* strains were inoculated into liquid low osmotic pressure MYA medium. After a 7-day shake-culture at 28°C and 250 rpm, the hyphae were collected by filtration on Whatmann paper. Then, the hyphae were inoculated on to solid low osmotic pressure MYA medium and cultured in the dark for 72 h at 28°C. At the time of 24 h, the spores (~10^8^) of WT (sexual spores) and the *ΔveA* deletion-type *A. cristatus* (only asexual spores were generated at this time) were collected and designated as WT and agamotype, respectively. At the time of 72 h, the spores mixed with conidia and ascospores were collected from *ΔveA* deletion-type and were designated the teleomorph. The spores of WT, the agamotype, and the teleomorph were stored at −80°C.

### Morphological observations

The morphology of spores from WT and *ΔveA* deletion-type *A. cristatus* after 24 and 72 h cultures were observed with an optical microscope (Olympus BX51; Tokyo, Japan).

### Protein extraction

Protein was extracted from the spores according to a protocol described previously [20]. Briefly, spores of the WT, agamotype, and teleomorph strains were collected from three biological cultures grown on low osmotic pressure solid medium, and washed in a phosphate buffer solution (pH 7.2). The spores’ samples were homogenized by vortexing in a solution containing 5 ml of Tris saturated phenol and 5 ml of extraction buffer (50 mM Tris/HCl, pH 8.6, 2% (SDS), 30% sucrose, and 2% 2-mercaptoethanol), incubated for 5 min on ice with vortexing, and centrifuged for 20 min at 6000 rpm and 4°C. After centrifugation, the upper layer with phenol was transferred to another centrifuge tube. Then, five volumes of ammonium acetate-methanol solution was added to precipitate the protein overnight at −20°C. After centrifugation for 20 min at 6000 rpm and 4°C, the supernatant was discarded. The precipitates were washed twice in 5 ml of methanol solution, then twice in 5 ml of acetone, followed by centrifugation for 20 min at 6000 rpm and 4°C each time. After vacuum cryodesiccation, the dried protein powder was collected and stored at −80°C. The protein powder was re-dissolved in lysis buffer (7 M urea, 2 M thiourea, 4% (g/ml) CHAPS, 65 mM DTT, and 0.01% (v/v) PMSF), incubated for 1 h on ice with vortexing every 15 min, and centrifuged for 1 h at 16100 rpm at 4°C to remove any insoluble material. The protein concentration of each sample was determined according to the Bradford method [21].

### 2-DE and image analysis

2-DE was performed according to a protocol reported previously by Zhou et al. (2011) [22], with a slight modification. Briefly, for isoelectric focussing (IEF), 450 μl IEF rehydration buffer (7 M urea, 2 M thiourea, 2% (g/ml) CHAPS, 1% (g/ml) DTT, 2% (g/ml) IPG buffer (pH 4–7), and 0.002% (g/ml) Bromophenol Blue) containing 1200 μg protein was loaded on to 24 cm (pH 4–7) Immobiline Dry Strips (GE Healthcare, Piscataway, NJ, U.S.A.) and separated using an Ettan IPGphor 3 Isoelectric Focusing System (GE Healthcare), according to the following parameters: 500 V for 1 h, 1000 V for 1 h, gradual increase in voltage up to 8000 V during 3 h, and then maintain 8000 V for ~7.5 h until total IEF voltage reached 60 kVh. After IEF, the IPG strip was equilibrated for 15 min in 10 ml reducing equilibration buffer (6 M urea, 50 mM Tris/HCl (pH 8.8), 30% (v/v) glycerol, 2% (g/ml) SDS, and 0.002% (g/ml) Bromophenol Blue) containing 2% (g/ml) DTT (freshly added when used), and then washed for another 15 min with equilibration buffer containing 2.5% (g/ml) iodoacetamide (freshly added). 2D SDS/PAGE (12.5% (w/v) homogeneous acrylamide gels (1 mm × 24 cm × 19 cm)) was performed using the Ettan DALT II system (Amersham Pharmacia, Buckinghamshire, U.K.) at 10°C and 2 W/gel for 45 min and then at 18 W/gel until the Bromophenol Blue reached the end of the gel. Protein markers within the range of 15–170 kDa were also loaded. After fixing the gels in fixation buffer (ethanol:glacial acetic acid:deionized water = 4.5:1:4.5) for 1 h, the spots on the 2-DE gels were detected by staining with Coomassie Brilliant Blue G-250 overnight and destained with deionized H_2_O.

Each gel was scanned (Powerlook 2100XL, UMAX) at 300 dpi, and an image analysis was performed using ImageMaster™ 2D Platinum 5.0 software (GE Healthcare). After automatic detection, the spots were detected by eye. The process of spot matching and normalization was performed manually to calculate spot intensity relative to the background (total intensity of spots presented on the 2-DE images) to reduce discrepancies during spot selection. Student’s *t*test and a significance level of 95% were selected to screen differentially expressed protein (DEPs) spots amongst the WT, agamotype, and teleomorph on triplicate gels. Spots that met the criteria of 1.5-fold change in intensity and *P*<0.05 were considered as DEPs, and were subjected to in-gel tryptic digestion.

### Protein enzymolysis and identification by MALDI-TOF/TOF-MS analysis

The equivalent DEP spots excised from the gels from the three repeat conditions were pooled and processed together. Protein enzymolysis of the DEPs with tryptase and the MALDI-TOF/TOF analysis were performed according to a protocol reported previously [22]. The tryptic peptides were analyzed on Ultraflex III TOF/TOF Analyzer (Bruker Daltonics Inc., Billerica, CA, U.S.A.). A UV laser with 200-Hz repetition rate, 355 nm wavelength, and 20 kV accelerating voltage was selected. The peptide mass fingerprint scan area was set to 700–3200 Da, and the optimal mass resolution rate was 1500 Da. Other parameters were set as stated by Liu et al. (2015) [23].

Flex analysis (Bruker Dalton) was applied to filter base peak and identify signal peak. The MS and the MS/MS spectral search was performed using BioTools (Bruker Daltonics) and MASCOT version 2.1 (Matrix Science, London, U.K.), according to the following parameters: NCBI non-redundant protein database (release date: 27 February, 2018; including 633912 proteins), and species restricted to *Aspergillus cristatus* first, then *Aspergillus*. The other parameters were as follows: peptide mass range 800–4000 Da; unrestricted for apparent isoelectric point and molecular weight; MS mass error range 50 ppm; MS-MS mass error range 0.5 Da; fixed modifications of carbamidomethylation (Cys); variable modifications of oxidation (met) and pyro-Glu (N-terminal Glu). Protein identification criteria were set as: at least two unique peptide matches, protein score of more than 95 and ≥95% confidence interval (C.I.%).

### Western blot analysis

A 25-μg aliquot of total protein from WT, agamotype, and teleomorph were separated by SDS/PAGE (12% gel) and electrotransferred to a PVDF membrane (Millipore, Bedford, MA, U.S.A.) using the Trans Blot system (Bio-Rad, Hercules, CA, U.S.A.) for the immunoblot analysis. Six polyclonal antibodies (Abcam, Cambridge, MA, U.S.A.) were selected, including anti-AAA ATPase (1:500), anti-heat shock protein (Hsp)70 (1:500), anti-SugarP isomerase (1:500), anti-40S ribosomal protein S0 (1:500), antivacuolar carboxypeptidase Cps1 (1:500), and anti-eukaryotic translation initiation factor 5A (1:500). Anti-β-tubulin (1:500) was used as the internal reference. After washing three times with PBST solution (100 mM Tris/HCl (pH 7.5), 0.9% (g/ml) NaCl, 0.1% (v/v) Tween-20), the PVDF membrane was incubated with a secondary horseradish peroxidase antibody conjugate for 1 h at room temperature. Then, the PVDF membrane was washed three times with PBST solution. Proteins were detected using the EasyBlot ECL kit (Thermo Scientific, Waltham, MA, U.S.A.), according to the manufacturer’s instructions. A Gel Doc XR system (Bio-Rad) was used for the membrane scanning and signal intensity analyses.

### RNA extraction and RT-qPCR

Total RNA was isolated using TRIzol reagent (Invitrogen) following the manufacturer’s instructions. The resultant RNA was applied in the reverse transcription reaction to obtain the first chain cDNA. Real-time qPCR reactions were carried out in a final volume of 25 μl, using SYBR Premix Ex Taq (TaKaRa), 0.4 mM of each primer, and 200 ng of cDNA template. The reaction parameters were set according to Ge et al. (2017) [5]. *β-tubulin* was used as the reference gene. The relative gene expression was evaluated using the comparative cycle threshold method [5]. At least three repeats were applied for each individual sample. The primers used presently were as follows: spot 3 (F: 5′-CCC CTA CTA CCA TCA CAA CAT CGC-3′, R: 5′- TCC ATT TCG CTT GTT TGC TCA CTG C-3′), spot 10 (F: 5′-CAG GTC CCT TCA GCC TTT CGG-3′, R: 5′-CTT GCT AAC TGG GTT TCC TTA ATA C-3′), spot 12 (F: 5′-ATA CTC GCT ATT CGT CGG TGC CTC GTC-3′, R: 5′-CCC ATA CCC TTC TTC AAA CAC TCA AAC TCG-3′), spot 13 (F: 5′-ACA TAA ACA CCC ACG CCC TCC TCT ACA CC-3′, R: 5′-CCA GAC GAA TAC GGA TGC GAG AAC GA-3′), spot 38 (F: 5′-CGT ATC ATC GCT ACC ATT GAC AAC CCG-3′, R: 5′-TAG CAG CAG CGA AAG CAG TGC CAG G-3′), spot 138 (F: 5′-AGC CTG TTG CGT ATC CCG TTG AGC-3′, R: 5′-GAG ACC GAG ATA CGG ATG ACC TGG C-3′), β-tubulin (F: 5′-TGT CCC TCG TGC CGT CCT CGT T-3′, R: 5′-ACT CCA TCT CGT CCA TAC CCT CAC C-3′).

### Statistical analysis

SPSS 19.0 statistical software (SPSS Inc., Chicago, IL, U.S.A.) was adopted for statistical analyses. Data were presented as mean ± S.E.M. One-way ANOVA was applied for data comparison, and significance was set at *P*<0.05.

## Results

### Morphological changes in the WT and *ΔveA* deletion-type *A. cristatus* strain

The morphology of WT and deletion-type *A. cristatus* strain was observed after 24 and 72 h of culture by optical microscopy. Eight sporangial structures were observed in the WT *A. cristatus* strain (Figure 1A,a), and asexual conidia were observed in *ΔveA* deletion-type after 24 h (Figure 1B,b), whereas some sexual ascospores appeared at 72 h, when the eight sporangial structures (cleistothecium) were observed in the deletion-type *A. cristatus* strain (Figure 1C,c,d). These results indicate that the *A. cristatus ΔveA* deletion mutant was recovered after prolonged culture in MYA medium.

### Protein profiles of the WT, agamotype, and teleomorph

To understand the role of VeA in *A. cristatus* spore sexual development at the molecular level, the protein profiles of the WT and *veA* mutant spores were compared. Total protein was extracted from the WT, agamotype, and teleomorph types, which were collected from 24 h cultures of the WT and *veA* deletion types, and from 72 h cultures of the *veA* deletion type strain grown on low osmotic pressure MYA solid medium. The proteins were separated by 2-DE. Totals of 1445 ± 20 (WT), 1542 ± 7 (agamotype), and 1542 ± 12 (teleomorph) protein spots were detected, and ~1357 spots were detected on all the gels (Supplementary Figure S1A,B). A total of 173 proteins spots with at least 1.5-fold change between the WT and agamotype/teleomorph strains were selected as DEPs (Supplementary Table S1).

### Identification of DEPs by MALDI-TOF-TOF

A MALDI-TOF-TOF analysis was applied to identify the DEPs mentioned above, and all 173 DEPs were successfully identified. The detailed information is presented in Supplementary Table S1. Amongst the identified proteins, 159 proteins with specific functions were successfully annotated in the current database. However, 14 proteins failed to annotate and were designated as unknown proteins (Supplementary Table S1). To acquire the possible functions of the unknown proteins, orthologs blasting was performed using their protein sequences against the non-redundant protein sequence database in NCBI (Blasttp). Orthologs with the highest similarity are presented in Supplementary Table S2. The results showed that all hits shared at least 59% sequence similarity, indicating similar functions between the unknown proteins and their orthologs.

Venn diagrams indicated that 84, 117, and 94 DEPs were detected in the WT, agamotype, and teleomorph, respectively (Figure 2). Approximately 9, 41, and 6 DEPs were considered unique proteins in the WT, agamotype, and teleomorph, respectively (Figure 2). Five DEPs were common to the WT, agamotype, and teleomorph (Figure 2). A pairwise comparison analysis revealed 34, 46, and 47 mutual DEPs between the WT and the agamotype, WT and the teleomorph, and the agamotype and teleomorph, respectively (Figure 2).

**Figure 2:** Venn diagram analysis of the DEPs isolated from the WT, agamotype, and teleomorph *A. cristatus*

Further analysis revealed that 103 and 66 DEPs were up-regulated in the agamotype and teleomorph, respectively (Table 1). However, 55 and 46 DEPs were down-regulated in the agamotype and teleomorph, respectively (Table 1). Amongst the up-regulated and down-regulated proteins, 44 and 21 DEPs were mutual, respectively (Table 1). Sixteen DEPs were up-regulated in the agamotype but down-regulated in the teleomorph, and thirteen DEPs were up-regulated in the teleomorph but down-regulated in the agamotype (Table 1).

**Table 1:** Number of differentially changed protein spots (DEPs) in the teleomorph and agamotype compared with WT

DEPs with different fold change	Teleomorph	Agamotype	Overlap
Up-regulated	66	103	44
Down-regulated	46	55	21
Up-regulated in agamotype but down-regulated in teleomorph			16
Up-regulated in teleomorph but down-regulated in agamotype			13

The experimental molecular weight (*Mr*) and isoelectric point (pI) values predicted by the protein ladders had an error deviation of approximately ±10% compared with the theoretical values. However, the observed *Mr* or *pI* values of some identified proteins were different from the theoretical values (Supplementary Table S1). An example is spot 1, which was an unknown protein. The experimental *Mr* of spot 1 was higher than the theoretical value (Supplementary Table S1), suggesting protein degradation. Moreover, some DEPs were identified as the same proteins, but showed different locations on 2-DE gels (Table 2). These results suggest post-translational modification or degradation of proteins after the *veA* gene was knocked out in *A. cristatus*.

**Table 2:** The same proteins with different location on the 2-DE gels

Spot number	Protein name	Experimental/theoretical		Accession	Coverage rate (%)
		Mass (kDa)	*pI*		
**Antioxidant and defense associated proteins**					
64	Putative glutathione S-transferase	23.84/25.87	6.91/6.46	gi|599156592	57
172	Putative glutathione S-transferase	24.21/25.87	6.63/6.46	gi|599156592	55
141	Superoxide dismutase [Cu-Zn]	13.21/16.03	6.55/6.14	gi|599159423	46
142	Superoxide dismutase [Cu-Zn]	12.99/16.03	6.59/6.14	gi|599159423	46
**Biosynthesis of secondary metabolites**					
70	Pigment biosynthesis protein brown 2	79.46/65.46	4.69/4.68	gi|599159066	21
148	Pigment biosynthesis protein brown 2	73.39/65.46	4.55/4.68	gi|599159066	18
**Carbon metabolism**					
44	Putative exo-β-1,3-glucanase	74.34/90.76	5.06/5.26	gi|599156967	11
147	Putative exo-β-1,3-glucanase	74.02/90.76	5.04/5.26	gi|599156967	11
76	Fructosyltransferase	68.36/56.69	4.44/4.53	gi|599151891	5
115	Fructosyltransferase	63.36/56.69	4.37/4.53	gi|599151891	15
152	Putative glucan 1,3-β-glucosidase A	39.93/45.92	4.62/4.81	gi|599155166	31
168	Putative glucan 1,3-β-glucosidase A	40.91/45.92	4.59/4.81	gi|599155166	27
79	Succinate dehydrogenase	63.04/71.38	5.84/6.16	gi|599155315	21
149	Succinate dehydrogenase	66.83/71.38	5.78/6.16	gi|599155315	33
140	Ribose/galactose isomerase	13.50/17.43	5.56/6.11	gi|599158499	40
145	Ribose/galactose isomerase	11.27/17.43	4.89/ 6.11	gi|599158499	51
**Energy metabolism**					
33	NAD(P)-binding protein	38.32/39.94	6.87/6.24	gi|599155554	30
34	NAD(P)-binding protein	38.16/39.94	6.65/6.24	gi|599155554	30
51	NAD(P)-binding protein	21.43/22.23	5.57/5.69	gi|599156176	23
52	NAD(P)-binding protein	21.37/22.23	5.81/5.69	gi|599156176	31
60	NADH-ubiquinone oxidoreductase 24-kDa subunit, mitochondrial	27.33/34.58	5.06/6.44	gi|599152277	27
111	NADH-ubiquinone oxidoreductase 24-kDa subunit, mitochondrial	28.22/34.58	5.05/6.44	gi|599152277	25
130	NAD(P)-binding protein	20.66/22.23	5.68/5.69	gi|599156176	37
131	NAD(P)-binding protein	20.91/22.23	5.91/5.69	gi|599156176	42
132	NAD(P)-binding protein	21.05/22.23	5.74/5.69	gi|599156176	49
133	NAD(P)-binding protein	20.82/22.23	5.85/5.69	gi|599156176	42
158	NAD(P)-binding protein	17.13/22.23	6.62/5.69	gi|599156176	43
162	NAD(P)-binding protein	13.00/22.23	4.79/5.69	gi|599156176	26
118	FAD-binding domain-containing protein	52.59/54.48	4.29/4.48	gi|599156179	19
136	FAD-binding domain-containing protein	18.78/22.26	5.88/5.72	gi|599156179	43
75	Putative NADH-ubiquinone oxidoreductase, subunit G	70.66/81.46	5.95/6.08	gi|599156753	30
77	Putative NADH-ubiquinone oxidoreductase, subunit G	67.69/81.46	5.67/5.47	gi|599156753	26
154	NAD(P)-binding protein	17.13/22.23	6.62/5.69	gi|599158621	31
155	NAD(P)-binding protein	13.00/22.23	4.79/5.69	gi|599158621	45
**Genetic information processing**					
36	Putative eukaryotic translation initiation factor 3 subunit EifCf	36.62/37.10	4.79/4.84	gi|599153195	15
101	Putative eukaryotic translation initiation factor 3 subunit EifCf	36.62/37.10	4.88/4.84	gi|599153195	17
40	Putative translation elongation factor EF-2 subunit	30.52/94.01	5.94/6.15	gi|599156428	11
41	Putative translation elongation factor EF-2 subunit	29.03/90.01	6.49/6.15	gi|599156428	14
55	Allergen Asp F3	12.13/18.63	4.98/5.30	gi|599157843	36
66	Allergen Asp F3	14.33/18.63	5.20/5.30	gi|599157843	12
144	Allergen Asp F3	11.94/18.63	5.12/5.30	gi|599157843	46
160	Allergen Asp F3	14.37/18.63	5.03/5.30	gi|599157843	17
53	Eukaryotic initiation factor 5a	16.27/51.62	5.91/5.85	gi|599159367	21
74	Eukaryotic initiation factor 5a	70.66/51.62	5.47/5.85	gi|599159367	21
80	Eukaryotic initiation factor 5a	63.92/51.62	6.16/5.85	gi|599159367	19
114	Eukaryotic initiation factor 5a	79.43/51.62	6.41/5.85	gi|599159367	24
138	Eukaryotic initiation factor 5a	15.91/51.62	5.86/5.85	gi|599159367	21
**Signal transduction**					
93	Rab GTPase activator	53.03/52.46	5.21/5.14	gi|599158509	35
151	Rab GTPase activator	48.81/52.46	5.11/5.14	gi|599158509	36
**Unknown**					
161	Hypothetical protein	13.05/14.77	4.44/4.77	gi|599159791	21
163	Hypothetical protein	12.19/14.77	4.60/4.77	gi|599159791	21
164	Hypothetical protein	12.07/14.77	4.43/4.77	gi|599159791	21
97	Hypothetical protein	48.71/47.23	5.63/5.35	gi|599159998	17
150	Hypothetical protein	49.79/47.23	5.52/5.35	gi|599159998	35

### Functional classification and subcellular localization of the DEPs in the WT, agamotype, and teleomorph

Based on a KEGG pathway analysis (http://www.kegg.jp/), all identified DEPs in *A. cristatus* were classified into 11 categories (Figure 3A,B and Supplementary Table S1), including genetic information processing (32.37%), carbon metabolism (16.18%), energy metabolism (15.61%), amino acid metabolism (10.40%), signal transduction (4.05%), biosynthesis of secondary metabolites (4.05%), antioxidant and defense (2.89%), lipid metabolism (3.47%), cytoskeletal-associated (1.73%), transport (1.16%), and unknown proteins (8.09%). The numbers of DEPs associated with these functions were largely different between the agamotype and teleomorph (Figure 3A,B). This finding suggests that protein expression levels were altered during sexual determination of spores after the *veA* gene was knocked out.

**Figure 3:** Functional classification and subcellular localization of the differentially expressed proteins (DEPs) in *A. cristatus* (A) Functional classification of the DEPs in the teleomorph; (B) functional classification of the DEPs in the agamotype; (C) subcellular localization of the DEPs in the teleomorph; (D) subcellular localization of the DEPs in the agamotype. Black and white bars represent the up- and down-regulated proteins, respectively. Abbreviations: cysk, cytoskeleton; cyto, cytoplasm; E.R., endoplasmic reticulum; extr, extracellular; mito, mitochondrial; nucl, nucleus; vacu, vacuole.

The online WoLF-PSORT (http://www.genscript.com/wolf-psort.html) and Euk-mPLoc 2.0 (http://www.csbio.sjtu.edu.cn/bioinf/euk-multi-2/#) tools were applied to predict the subcellular localization of all identified DEPs using the DEP protein sequences. The results indicated that the majority of the identified DEPs in *A. cristatus* were localized in the cytoplasm, mitochondria, nucleus, and extracellular matrix (Figure 3C,D). Interestingly, 29 proteins are located in nucleus for agamotype, 20 of them were up-regulated, and mostly associated with the genetic information processing (Figure 3D and Supplementary Table S1), which indicated that the process of transcription, translation, protein folding, and degradation were interfered after the *veA* deletion, thereafter, disturbed the spores gender of *A. cristatus*. Further analysis was performed in the following sections.

### Validation of DEPs by Western blot and RT-qPCR analysis

To confirm the reliability of the DEPs identified in the 2-DE analysis, six DEPs in *A. cristatus*, including AAA ATPase (spot 3), Hsp70 (spot 10), SugarP isomerase (spot 12), vacuolar carboxypeptidase Cps1 (spot 13), 40S ribosomal protein S0 (spot 38), and eukaryotic translation initiation factor 5A (spot 138), were selected for Western blot and **RT-qPCR** analysis. β-tubulin was used as the internal protein reference (Figures 4A and 5A). The results revealed that the changed abundance pattern of the DEPs determined by the Western blot and RT-qPCR analysis was in accordance with the trends detected by 2-DE (Figures 4A,B and 5A,B), suggesting high reliability of the proteomics results.

**Figure 4:** Comparison of the abundance of differentially changed proteins determined by Western blot and 2-DE analyses (**A**) Western blot analysis results; (**B**) The relative 2-DE analyses results. The spot identities correspond to those in Supplementary Table S1.

**Figure 5:** Gene expression analysis by RT-PCR and RT-qPCR The log_1.5_ values of the ratio of agamotype or teleomorph to the control sample are plotted. (**A**) RT-PCR results of spots 3, 10, 12, 13, 38, and 138. (**B**) RT-qPCR results of spots 3, 10, 12, 13, 38, and 138.

## Discussion

### The *veA* deletion-induced change in spores gender were determined by signal transduction associated proteins in *A. cristatus*

Previous studies in *A. nidulans* revealed that at least three stages occur in the asexual reproductive cycle, starting with the perception of induction signals during the growth phase, initiation of various developmental and metabolism pathways, and the developmentally modulated events executed to generate sporulation [24]. Disruption of Ser-Thr-rich glycosyl-phosphatidyl-inositol-anchored membrane proteins (GPI-APs, spot 139) affect ascospore cell wall formation in yeasts *Saccharomyces cerevisiae SPS2* and *Schizosaccharomyces pombe meu10* families, and resulted in a conidium phenotype [25,26]. Takada et al. (2010) [27] found that deletion of Ecm33 (a GPI-AP) was involved in the hyperactivation of Pmk1-MAPK signaling pathway by affecting Ca^2+^ homeostasis in fission yeast. While Pmk1-MAPK signaling plays a role in conidiation of *Magnaporthe oryzae* [28]. Coincidently, the expression levels of GPI-APs in the WT, agamotype, and teleomorph were 40.11 ± 10.69, 0.00, and 12.88 ± 10.67, respectively (Figure 6 and Supplementary Table S1). It is implied that the deletion of GPI-APs in the *A. cristatus veA* deletion mutant (agamotype) resulted in the production of conidia through affecting ascospore cell wall formation, which was involved in Pmk1-MAPK signaling.

**Figure 6:** DEPs associated with signal transduction in *A. cristatus* All protein spots are enlarged from Supplementary Figure S1 and protein intensity values are from Supplementary Table S1. Error bars represent S.D. (*n*=3).

Protein phosphatase 2A (PP2A) regulatory subunits mediate specific substrates associated with various signaling pathways by reversible protein phosphorylation to control different processes, and are necessary for hyphal growth, conidiation, and self-fertilization, by maintaining normal level of PP2A activity [29]. Similar to PP2A, protein phosphatase 2C (PP2C) is a class of Ser/Thr phosphatases that play vital roles in functional processes in fungi, such as negatively regulating cell growth and cellular stress signaling, counteracting the function of MAPKK WIS1 in osmoregulation, and sequentially activating and inactivating cyclin-dependent protein kinases during growth [30]. However, the difference between PP2A and PP2C lies in functional specificity achieved by encoding multiple PP2C isoforms not usually associated with regulatory subunits [31]. Currently, a protein phosphatase PP2A regulatory subunit A (spot 71) and a PP2C protein (spot 81) were up-regulated in the agamotype but relatively down-regulated in teleomorph compared with agamotype (Supplementary Table S1), suggesting possible function of PP2A regulatory subunit A and PP2C in conidiation of the *A. cristatus veA* deletion mutant at the differentiation stage under low osmotic stress.

Totally, it is speculated that the deletion of *veA* resulted in the disturbance of signaling pathways, including Pmk1-MAPK and Ser/Thr phosphatase signalings. Thereafter, asexual spores were produced in *A. cristatus veA* deletion mutant.

### Changes in genetic information processing-associated and amino acid metabolism-associated proteins

The VeA protein is localized in the nucleus where it regulates sporulation by interacting with other regulatory proteins, such as FphA, LreA, LaeA, and VelB, leading to transcriptional regulation of genes associated with induction/repression of sexual spore development [14,15]. Currently, after the deletion of *veA* gene in *A. cristatus*, a total of 56 DEPs were involved in genetic information processing (Supplementary Table S1 and Figure 7A) and were classified into three groups of transcription associated, translation associated, and protein processing associated (folding and degradation).

**Figure 7:** Hierarchical clustering of DEPs associated with genetic information processing and amino acid metabolism in *A. cristatus*. (A) protein spots associated with genetic information processing; (B) protein spots associated with amino acid metabolism. A hierarchical cluster analysis was conducted using the Genesis software package version 8.2 1.7.6 (Graz University of Technology, Austria, http://genome.tugraz.at/genesisclient/genesisclient_download.shtml) and the log_1.5_-transformed values of fold-change ratios were adopted. Protein spot identities correspond to those in Supplementary Table S1.

Nine DEPs were associated with the synthesis of nucleotides, which also were categorized in the process of transcription (Supplementary Table S1 and Figure 7A), including purine biosynthesis involved proteins GMP synthetase (GMPS, spot 16) [32] and adenylyl-sulphate kinase (ASK, spot 61) [33]. Both of them were decreased in the agamotype but increased in the teleomorph (Supplementary Table S1 and Figure 7A). However, the purine degradation associated protein Uricase (spot 109) [34] was up-regulated in the agamotype but did not change in the teleomorph. These results indicated that purine synthesis was enhanced in the *veA* deletion mutant of *A. cristatus*.

Carbamoyl-phosphate synthase arginine-specific large chain (CMPL, spot 56), dUTPase (spot 67), and uracil phosphoribosyltransferase furA (UraPRT-furA, spot 173) are pyrimidine metabolism-associated proteins. CMPL plays a role in pyrimidine biosynthesis and participates in the arginine synthetic pathway [35]. dUTPase hydrolyzes dUTP to dUMP and provides a substrate for synthesis of TTP [36], and was up-regulated in the agamotype and teleomorph (Figure 7A). However, expression of UraPRT-furA was suppressed both in the agamotype and teleomorph (Figure 7A), which catalyzes the first step of UMP biosynthesis [37], indicating a decrease in dUMP synthesis.

A total of 20 proteins were involved in the process of translation (Figure 7A). Amongst them, 12 proteins were up-regulated in the agamotype, but down-regulated in the teleomorph compared with the agamotype, including RNA recognition and binding proteins, translation initiation factors and elongation factors (Figure 7A and Supplementary Table S1). These results suggest that protein synthesis was mainly enhanced after deletion of the *veA* gene in *A. cristatus* under low osmotic stress, but this condition changed when culture time was prolonged and most of these protein profiles were recovered.

Twenty-seven DEPs were protein processing-associated proteins. These proteins were separately classified into protein folding (chaperone) and protein degradation groups according to their biological functions. Eleven proteins functioned as chaperones; seven increased in the agamotype, but decreased in the teleomorph (compared with the agamotype), and three of the chaperones increased in the teleomorph but decreased in the agamotype (Figure 7A). It has been reported that suppressing *HSP90* leads to defects in asexual sporulation in *Fusarium graminearum*, and this gene is involved in repressing the conidiation-specific genes *BRLA, WETA, STUA, HTF1, REN1*, and *ABAA* [38], indicating the vital role of HSP90 in asexual sporulation. Conicidently, the expression of HSP90 (spot 72) was increased, implied enhanced asexual sporulation in the agamotype of *A. cristatus* (Figure 7A).

Of the 16 degradation-associated proteins, the expression of 10 increased and that of 6 decreased in the agamotype (Figure 7A). One kind of degradation-associated protein, hydrolytic enzymes (proteases), play a critical role in response to the host environment of *A. fumigatus* [39]. Only 15% protease activity has been detected in the *veA* deletion mutant compared with the WT strain of *A. fumigatus* [12]. In contrast, the expression levels of the hydrolytic-associated proteins identified here were mainly enhanced (Figure 7A). However, deletion of *veA* in *A. fumigatus* resulted in reduced production of conidia [12]. Therefore, we surmized that the sexual sporulation-associated proteins were depressed because of protein degradation, whereas asexual spore production was enhanced in *A. cristatus*.

Amino acids are the basic constituent of functional proteins. Sulphur-containing proteins are widely distributed in living organisms and play important physiological roles, including asexual and sexual spore determination [40]. The initiation of sulphate assimilation in yeast is the beginning of adenosine 5′-phosphosulphate production by phosphorylation and 3(2),5-bisphosphate nucleotidase, which is encoded by the *HAL2* gene, and is involved in the methionine biosynthetic [41] and homocysteine synthase alternative cysteine synthetic pathways [42]. Here, four proteins were involved in the sulphur amino acid metabolism, including homocysteine synthase (spot 23) and assimilatory sulphite reductase (spot 57), which are related to cysteine synthesis, and S-adenosyl-l-methionine-dependent methyltransferase (spot 26) and 3(2),5-bisphosphate nucleotidase HAL2 (spot 30), which are involved in methionine synthesis. These proteins all showed increased expression in the agamotype, but decreased expression in the teleomorph compared with the agamotype (Supplementary Table S1 and Figure 7B). Adomet-Mtase S-adenosylmethionine-dependent methyltransferase (MoIlv6) plays a vital role in leucine, isoleucine, and valine biosynthesis. Knockdown of *MoIlv6* in *M. oryzae* results in retarded growth, reduced conidiation, and invasive hyphal growth [43]. Coincidently, two valine, leucine, and isoleucine biosynthesis-involved proteins were detected in the present study, including dihydroxy-acid dehydratase (spot 15) [44] and 2-isopropylmalate synthase (spot 73) [45], which were both up-regulated in the agamotype but down-regulated in the teleomorph compared with the agamotype (Supplementary Table S1 and Figure 7B), indicating enhanced biosynthesis of valine, leucine, and isoleucine in the agamotype. This result suggests that the enhanced asexual sporulation in the agamotype was correlated with enhanced leucine, isoleucine, and valine biosynthesis. Four DEPs were arginine metabolism-associated and increased in expression in the agamotype but decreased expression in the teleomorph compared with the agamotype (Supplementary Table S1 and Figure 7B). These proteins were argininosuccinate synthase (spot 22) [46], acetylornithine and succinylornithine aminotransferase (spot 24) [47], putative l-ornithine aminotransferase Car2 (spot 25) [48], and spermidine synthase (spot 159) [49]. One arginine metabolism-associated protein (spot 121, peptidyl-arginine deiminase domain protein [50]), decreased in expression in the agamotype but increased expression in the teleomorph compared with the agamotype. The arginine biosynthetic bifunctional protein ArgJ β-chain (spot 171) [51] did not change significantly in the agamotype but decreased in the teleomorph (Supplementary Table S1 and Figure 7B). These results suggest that arginine biosynthesis was promoted in the agamotype but relatively recovered in the teleomorph. *Clostridium botulinum* cultured on medium without arginine does not undergo proper sporogenesis until the arginine concentration increases to the normal level [52], indicating a vital role for arginine in sporulation. Three PLP-dependent transferases (spots 19, 83, and 84) associated with the biosynthesis of alanine, aspartate, and glutamate [53] showed enhanced expression in the agamotype but decreased expression in the teleomorph compared with the agamotype (Supplementary Table S1 and Figure 7B). The putative phosphoribosyl-AMP cyclohydrolase (spot 59) involved in histidine metabolism [53] and the putative anthranilate synthase multifunctional protein TrpC (spot 69) involved in phenylalanine, tyrosine, and tryptophan biosynthesis [54] both increased in expression in the agamotype but decreased in the teleomorph compared with the agamotype (Supplementary Table S1 and Figure 7B). A putative dimethylallyl tryptophan synthase (spot 46) associated with tryptophan synthesis [55] showed decreased expression in the agamotype but increased expression in the teleomorph compared with the agamotype (Supplementary Table S1 and Figure 7B). These results reveal that the VeA protein participates in several amino acid metabolic pathways. Similarly, the comparative proteomics analysis of the *Morgs1-8* (G-protein signaling associated) deletion mutant reveals a distinct and specific role in the regulation of amino acid metabolism of each MoRgs protein in *M. oryzae* [18]. As each amino acid-associated protein was distinct in the agamotype and teleomorph, it may also be true that amino acid metabolism was recovered by other regulatory proteins when culture time was prolonged in the *A. cristatus veA* mutant under low osmotic conditions.

Concludingly, the increased expression of HSP90, protein degradation associated proteins, sulphur-containing amino acid biosynthesis associated proteins, valine, leucine, isoleucine and arginine biosynthesis-involved proteins may have resulted in the production of conidia in agamotype.

### Carbon metabolism and energy metabolism-associated proteins change in the *A. cristatus* agamotype and teleomorph

Glucose catabolic pathways (carbon metabolism) can be distinctly divided into glycolysis (also called the Embden–Meyerhof pathway), tricarboxylic acid (TCA) cycle, and the pentose phosphate pathway (PPP). These processes produce energy for normal growth and differentiation, besides, TCA cycle also produce precursors for biosynthetic pathways and PPP produce reducing compounds, such as NADPH, for biosynthesis [23,56]. In the present study, 15 DEPs were associated with glycolysis, eight were involved in the TCA cycle and four were involved in the PPP in the *A. cristatus veA* deletion mutant. Ten of fifteen DEPs related to glycolysis were significantly up-regulated in the agamotype, whereas they decreased in the teleomorph compared with the agamotype. Three DEPs (spots 44, 153, and 168) did not change significantly in the agamotype but increased in the teleomorph, and only two DEPs (spots 115 and 165) were down-regulated in the agamotype (Figure 8A), suggesting that glycolysis is prominent in the agamotype. This finding verifies that the primary metabolism may have been modulated to establish a new homeostasis after the *veA* gene was silenced in *A. cristatus*. Similar with the changing pattern of glycolysis, expression of most of the TCA cycle-associated proteins (seven of eight DEPs) in the agamotype increased, whereas they decreased in the teleomorph compared with the agamotype, and only one protein decreased in the agamotype (spot 124). These results suggest that enhanced energy production was obtained through glycolysis and the TCA cycle in the agamotype, and that the biosynthetic pathways may have also been enhanced by producing precursors during the TCA cycle, but the teleomorph showed an opposite pattern. In contrast, expression of the four PPP-associated proteins all decreased in the agamotype but increased in the teleomorph relative to the agamotype. Two GroES-like proteins (spots 47 and 123) and two ribose/galactose isomerases (spots 140 and 145) (Figure 8A) indicated suppression of anabolism through the PPP in the agamotype.

**Figure 8:** Hierarchical clustering of DEPs associated with carbon metabolism and energy metabolism in *A. cristatus* (A) protein spots associated with carbon metabolism; (B) protein spots associated with energy metabolism.

Changes in carbon metabolism are tightly correlated with energy metabolism in live cells [23,56]. A total of 27 DEPs related to energy metabolism were detected, including one ATP-associated protein (spot 3), two FAD-binding proteins (spots 118 and 136), five NADH associated proteins (spots 65, 70, 77, 111, and 112) and 19 NAD(P)-binding proteins (spots 33, 34, 49, 51, 52, 85, 110, 126, 130, 131, 132, 133, 134, 137, 154, 155, 158, 162, and 170) (Figure 8B). Expression of the ATP-associated protein AAA ATPase (spot 3) and all five NADH-associated proteins (spots 60, 75, 77, 111, and 112) increased in the agamotype, whereas they decreased in the teleomorph relative to the agamotype (Figure 8B). Expression of both FAD binding proteins (spots 118 and 136) and 11 of 19 NAD(P)-binding proteins decreased in the agamotype but increased in the teleomorph compared with the agamotype (spots 49, 51, 52, 126, 130, 131, 132, 133, 134, 137, and 170). Expression of 3 of 19 NAD(P)-binding proteins did not change significantly in the agamotype but expression increased in the teleomorph compared with the agamotype (spots 34, 158, and 162). Expression of only 5 of 19 NAD(P)-binding proteins increased in the agamotype but decreased in the teleomorph compared with the agamotype (spots 33, 85, 110, 154, and 155) (Figure 8B). These results suggest that the energy compounds produced from carbon metabolic pathways were mainly in the form of ATP and NADH in the agamotype, whereas they were NADPH and FAD in the teleomorph.

Glycolysis and the TCA cycle were enhanced, while the PPP was suppressed in the agamotype, in conjunction with promoted catabolism and depressed anabolism in the agamotype. However, glycolysis, the TCA cycle, and PPP-associated proteins changed in different ways in the teleomorph. The energy compounds produced in the agamotype were mainly ATP and NADH, whereas they were NADPH and FAD in the teleomorph.

### Lipid metabolism-associated proteins are mainly repressed in the agamotype

Six DEPs detected in the *A. cristatus veA* deletion mutant were involved in lipid metabolism (Figure 9), including decreased expression of the phytanoyl-CoA dioxygenase family protein (spot 39), fatty acid amide hydrolase (FAAH, spot 117), CRAL/TRIO domain-containing protein (spot 119), and CoA-dependent acyltransferase (spot 120) in the agamotype; expression of these increased in the teleomorph. Expression of the other two lipid-associated proteins, such as sterol 24-C-methyltransferase (spot 35) and Sec14p-like lipid-binding (spot 102), increased in the agamotype but decreased in the teleomorph. Phytanoyl-CoA dioxygenase (spot 39) plays a role in fatty acid degradation by α-oxidizing branched chain fatty acids (e.g. phytanic acid) in peroxisomes. A putative fatty acid dioxygenase PpoA, regulated by VeA and the COP9 signalosome participates in the biosynthesis of oxylipin psiBα and is critical for balancing anamorph and teleomorph development in *A. nidulans*. The deletion mutant without the *ppoA* gene exhibited a significant decrease in the expression level of psiBα and an increase in the ratio of asexual to sexual spores, whereas forced expression of PpoA presented contrasting results [57]. These data indicate an important role for fatty acid dioxygenase integrating mitotic and meiotic spore development. Furthermore, a proteomics analysis of *Penicillium chrysogenum* revealed the role of phytanoyl-CoA dioxygenase in the biosynthesis of penicillin [58]. FAAH possesses esterase and amidase activity *in vitro* and plays a principal role in catabolism of bioactive lipids, including anandamide and oleamide [59]. These bioactive lipids are categorized as fatty acid amides that modulate the interaction between fungi and their host plants [60]. The CRAL/TRIO domain-containing protein (spot 119), the Sec14p-like lipid-binding protein (spot 102), and CoA-dependent acyltransferase (spot 120) are all required for phospholipid transfer activity and are associated with G-protein β/γ subunits, which means they play a role in a signaling pathway [61]. Expression of these mainly decreased in the agamotype but increased in the teleomorph, except Sec14p-like lipid-binding protein, indicating that VeA positively regulates the activity of phospholipid metabolism-associated proteins.

**Figure 9:** Hierarchical clustering of DEPs associated with antioxidation and biosynthesis of secondary metabolic, cytoskeletal, lipid metabolic, and transport proteins in *A. cristatus*

### Proteins involved in the biosynthesis of secondary metabolites are mainly enhanced in the agamotype

VeA regulates the biosynthesis of many secondary metabolites in filamentous fungi, including positive regulation of ochratoxin A, which is a nephrotoxic, teratogenic, and immunotoxic mycotoxin in *A. carbonarius* [62]; however, VeA negatively regulates synthesis of other secondary metabolites, including kojic acid, oryzachlorin, and asperfuran in *A. flavus* [63]. Seven DEPs were associated with biosynthesis of many secondary metabolites in the *A. cristatus veA* deletion mutant. Expression of all these proteins increased in the agamotype but decreased in the teleomorph compared with the agamotype, except cytochrome P450 (spot 135, Figure 9), a class of proteins containing heme as a cofactor that mediate diverse cellular/metabolic processes, including secondary metabolism in fungus, such as biosynthesis of trichothecene [64], butenolide [65], culmorin [66] and ergostero [67] in the filamentous fungi *F. graminearum*. It has been reported that some *F. graminearum CYP450* gene deletion mutants show reduced conidia production, while some other *CYP450* gene deletion mutants exhibit defects in sexual reproduction [68]. Overall, decreased expression of CYP450 in the *A. cristatus veA* deletion mutant resulted in reduced production of trichothecene, butenolide, culmorin, and ergosterol, disrupting the balance between asexual and sexual sporulation.

1,3,6,8-Tetrahydroxynaphthalene reductase (T4HR, spot 6) expression increased in the agamotype but decreased in the teleomorph (Figure 9). T4HR converts 1,3,6,8-THN into scytalone during melanin biosynthesis in *Bipolaris oryzae* [69], whereas 1,3,6,8-tetrahydroxynaphthalene synthase (T4HS) spontaneously oxidizes 1,3,6,8-THN to form flaviolin [70]. Disruption of the *T4HR1* gene results in colonies of a vivid orange color, whereas a muddy orange color was observed in the WT, indicating that the shunt products flaviolin and 3,3-biflabiolin accumulate in the *T4HR1* deletion mutant because conversion of T4HN into scytalone was completely suppressed [71]. Pigment biosynthesis protein brown 2 (spots 70 and 148) is a cupredoxin domain protein that functions similar to Abr2 in *A. fumigatus*. Abr2 is involved in conidial pigment biosynthesis in *A. fumigatus* by the accumulation of scytalone and flaviolin in different *Abr2* gene deletion mutants through the DHN-melanin pathway [72,73]. In accordance with the T4HN findings from *B. oryzae* and Abr2 from *A. fumigatus*, deleting *veA* enhanced T4HR and pigment biosynthesis protein brown 2 in *A. cristatus* and forced the formation of scytalone and/or flaviolin, which ultimately changed the color of the colony (Figure 1).

The aromatic prenyltransferase (spot 9) catalyzed C-prenylation of aromatic substrates in secondary metabolism, which involves biosynthesis of pulvinone, flaviolin, and 4-hydroxybenzoic acid in *A. terreus* [74] or indole derivatives in *A. fumigatus* and *Neosartorya fischeri* [75]. The aflatoxin B1 aldehyde reductase-like protein (spot 105) participates in biodegradation and metabolism of aflatoxin B1 [76]. Nicotinate-nucleotide pyrophosphorylase (spot 107) is involved in the production of nicotinic acid mononucleotide [77]. The expression of all these proteins increased in the agamotype but decreased in the teleomorph (Figure 9) of the *A. cristatus veA* deletion mutant, suggesting that VeA may positively regulate biosynthesis of pulvinone, flaviolin, 4-hydroxybenzoic acid, and nicotinic acid mononucleotide, but negatively regulate the biosynthesis of aflatoxin B1 in *A. cristatus*.

Taken together, these results suggest that *veA* deletion affects pigmentation and biosynthesis of secondary metabolites in *A. cristatus*.

### Cytoskeletal associated proteins are enhanced in the agamotype and involved in conidiophore development

The formation of conidiophores in a fungal colony starts with the growth of a conidiophore stalk that elongates by apical extension of an aerial hyphal branch. When the stalk gains a height of 100 μm, the apical extension and polar growth of the germ tube stops, and the tip begins to swell to form the conidiophore vesicle. Multiple nuclei aligned around outside the vesicle undergo several synchronized mitoses as the conidiophore stalk elongates and the vesicle expands, and shapes a structure called the metulae. In the succession to polar growth by metular budding, phialides with a layer of ~120 uninucleate sterigmata produce the end of the metula, and the mature conidia are produced from the phialides [24]. Actins play an extremely pivotal role during apical extension, polar growth, and mitosis/meiosis by depolymerizing and/or repolymerizing to form microfilaments [78]. Here, four microfilament-associated proteins, the actin-related protein 4 (spot 20), Ca^2+^-binding actin-bundling protein fimbrin/plastin (spot 78), the actin depolymerizing protein (spot 99), and the BAR domain protein (spot 100, actin cytoskeleton organization associated) were detected and their expression all increased in the agamotype but decreased in the teleomorph compared with the agamotype, indicating a critical role in asexual sporulation of the *A. cristatus veA* deletion mutant.

## Conclusion

In the present study, morphological changes and proteomic alterations were detected in the agamotype and teleomorph of the *A. cristatus veA* deletion mutant to reveal the regulatory mechanism of VeA during asexual sporulation under hypotonic conditions. The morphological data indicate that only conidia were produced by the *A. cristatus veA* deletion mutant after a 24-h culture in hypotonic medium, where only the WT should produce ascospores. However, both sexual and asexual spores were generated after 72 h in the *veA* deletion mutant, but only sexual spores were generated in the WT. A comparative proteomics analysis identified 173 DEPs in the agamotype and teleomorph of the *A. cristatus veA* deletion mutant. The DEPs identified with known functions were classified into 11 categories of signal transduction, genetic information processing, amino acid metabolism, carbon metabolism, energy metabolism, signal transduction-associated proteins, lipid metabolism, and biosynthesis of secondary metabolites and cytoskeletal and transport proteins. Further analysis revealed that the changed expression pattern of Pmk1-MAPK and Ser/Thr phosphatase signaling proteins, HSP90, protein degradation associated proteins, sulphur-containing amino acid biosynthesis associated proteins, valine, leucine, isoleucine and arginine biosynthesis-involved proteins, CYP450 and cytoskeletal formation associated proteins were involved in the production of conidia in agamotype of *A. cristatus*. Furthermore, the deletion of *veA* in *A. cristatus* resulted in disturbed process of transcription, translation, protein folding, amino acid metabolism, and secondary metabolism. The carbohydrate and energy metabolism were also greatly changed, which lied in the suppression of anabolism through PPP but promotion of catabolism through glycolysis and TCA cycle. The energy compounds produced in the agamotype were mainly ATP and NADH, whereas they were NADPH and FAD in the teleomorph. These results will contribute to the existing knowledge on the complexity of the VeA regulatory system that functions in sporulation of filamentous fungi. Our results will provide a framework for further functional studies on each of the identified proteins.

## Supporting information

**supplementary Figures:** 

**Supplemental Table 1:** Differentially changed proteins in the Wild type, agamotype and teleomorph of Aspergillus cristatus identified by MALDI-TOF-TOF

## Abbreviations

CMPL: carbamoyl-phosphate synthase arginine-specific large chain
2-DE: 2D electrophoresis
DEP: differentially expressed protein
FAAH: fatty acid amide hydrolase
GPI-AP: glycosyl-phosphatidyl-inositol-anchored membrane protein
Hsp: heat shock protein
IEF: isoelectric focussing
*Mr*: experimental molecular weight
*pI*: isoelectric point
PPP: pentose phosphate pathway
PP2A: protein phosphatase 2A
PP2C: protein phosphatase 2C
TCA: tricarboxylic acid
T4HR: 1,3,6,8-tetrahydroxynaphthalene reductase
UraPRT-furA: uracil phosphoribosyltransferase furA
WT: wild-type
